# Real-Time Gait Intention Recognition for Active Control of Unilateral Knee Exoskeleton

**DOI:** 10.1155/2024/9426782

**Published:** 2024-11-13

**Authors:** Ziwei Zhang, Xuefeng Cai, Minbo Zhang, Wuxiong Chen, Yijie Chen, Pu Wang

**Affiliations:** ^1^Rehabilitation Medicine Department, The Seventh Affiliated Hospital of Sun Yat-Sen Univerity, Shenzhen 518000, China; ^2^Shenzhen Chwishay Intelligent Tech Co., Ltd., Shenzhen 518000, China; ^3^Rehabilitation Medicine Department, Shanghai Health Rehabilitation Hospital, Shanghai 200000, China; ^4^Department of Rehabilitation, Sichuan Provincial People's Hospital, Chengdu 610072, China

## Abstract

Real-time gait estimation is important for the synchrony control of robotic exoskeleton to provide walking assistance. However, for stroke patients with hemiplegic paralysis, the gait pattern is very complex. Accurate and timely gait intention recognition is therefore difficult. To achieve human–robot synchrony control for an unilateral knee exoskeleton, a gait intention recognizer coupling the adaptive frequency oscillator (AFO) and back propagation neural networks (BPNN) is proposed in this paper. The BPNN is trained with gait data of healthy subjects and stroke patients to improve the accuracy of recognized gait pattern, which is then imported into flexible interaction module to provide appropriate assistance. To evaluate the performance of gait intention recognition, three stroke patients were recruited to conduct level ground walking tests. The kinematic and biomechanical data were captured in each test and processed for the evaluation. Experimental results demonstrate the effectiveness of gait intention recognition and movement assistance.

## 1. Introduction

Robotic rehabilitation presents a promising solution to the situation of fast-growing number of stroke patients and predicted shortage of professional rehabilitation therapists [1, 2, 3]. Heretofore, lower limb exoskeletons focusing on different joints have been widely used for gait rehabilitation. Compared with bilateral exoskeletons for spinal cord injury patients, unilateral exoskeletons are more beneficial to stroke survivors with hemiplegic paralysis. Therefore, unilateral exoskeletons have attracted more attention over the previous decades, in which the knee joint is the major assistive target for its importance in accomplishing bipedal ambulation in daily life [4, 5, 6, 7, 8].

Offering patients with proper assistance, which requires an optimal control strategy, is one of the major concerns in designing unilateral knee exoskeleton to maximize the rehabilitation effect [9]. In state-of-art studies, control strategies, such as position control, torque control, and impedance control, have been widely applied to rehabilitation robots [10]. For gait rehabilitation, the involving motion intention control strategy, which provides appropriate force and safe interaction, remains challenging. The complexity of human motion suggests the need of a robust perception system, and the perception of gait is the priority for lower limb exoskeleton. Gait is a periodic motion with specific frequency, phase, and amplitude for each individual. Therefore, the perception of gait means recognition of these characters.

To realize accurate prediction, the sensing systems and algorithms are designed to interpret the gait signals. Therefore, sensors play a significant role in measuring, classification, and control of exoskeletons. Bioelectrical sensors, such as surface electromyography (sEMG) and electroencephalograph (EEG), have been commonly used in motion perception [11, 12, 13, 14, 15]. However, due to relatively low amplitude, these biosignals can be easily interfered by the electrodeposition, electrical noise, and surrounding conditions [16]. In contrast, mechanical sensors, such as the inertial measurement unit (IMU), are more robust and easily embedded with rehabilitation robots [17, 18]. Owing to the precision and easy integration of mechanical sensors, the IMUs are utilized for gait recognition.

For gait recognition, one of the approach to simplify the task is by representing the cycle as a finite set of states and transitions between them. Therefore, the finite state machine (FSM) is widely used for discrete gait phase. Wang et al. [19] proposed to optimize the parameters in the FSM states and feedback laws, with the objectives of naturalness and controllability of the generated motion. Apart from single gait phase recognition, FSM is also used for different gait tasks. Jang et al. [20] designed an assistance strategy based on FSM to recognize stair ascent gait phase. The entire task was decomposed into four states, and the states were recognized by information from mechanical sensors. Similar work was also conducted in [21] to provide assistance in different terrain. Although FSM is effective in discrete states recognition, the discrete gait event could only provide rough assist torque, which is not conductive to the improvement of assist efficiency [22].

The adaptive frequency oscillators (AFO) provides an idea to estimate the gait continuously and has been a popular exoskeleton control architecture for its fewer sensor requirements and strong robustness [23, 24, 25, 26, 27, 28, 29, 30]. AFO was originated from the dynamic Hebbian learning rule in the nonlinear oscillator, which was first proposed by Righetti et al. [31] to synchronize with a periodic or pseudoperiodic signal. Then it was applied to human–robot synchrony control, where the AFO was utilized to extract periodic motion features and predict assistive pattern. The gait phase is the major concern of the intention estimation and assistive control. Though the adaptive law is effective in frequency and phase learning, the results show poor performance on the amplitude tracking [32]. The AFO-based control strategy was mainly applied to performance augmentation for normal gait pattern. For stroke patients with hemiplegic paralysis, the gait pattern is complex, and gait parameters could vary with cycles. Accurate recognition of phase and amplitude is necessary for providing appropriate assistance without damages. In addition, the learning process is time-consuming for AFO to obtain parameters from several similar gait cycles. Timely recognition is also the key requirement for active control system.

To address these issues, the AFO cascaded with back propagation neural networks (BPNN) is proposed in this paper to recognize the gait pattern for an unilateral knee exoskeleton gait rehabilitation training robot (GRTR). AFO is responsible for learning and predicting the frequency and phase of gait pattern from hip joint. Based on the recognition of hip joint motion, the BPNN is utilized to realize the accurate recognition of the target knee joint. The gait data for training BPNN was collected from both healthy subjects and stroke patients. The specially trained BPNN is therefore cascaded to improve gait frequency, phase, and amplitude recognition performance for knee joint. The recognized motion intention is then imported to flexible interaction module to generate corresponding assisting torque.

The rest of this paper is organized as follows: Section 2 describes the methods including GRTR design and active control system especially the intention recognition in detail.  Section 3 contains the experiments to verify the performance of the proposed gait intention recognition for active control. Discussion and conclusion are presented in Sections 4 and 5.

## 2. Materials and Methods

### 2.1. Unilateral Knee Exoskeleton

The knee exoskeleton GRTR weighs about 2 kg and has the advantage of convenient wearing, as is illustrated in Figure 1(a). The GRTR mainly consists of a powered knee joint and connecting mechanisms (Figure 1(b)). The powered joint is implemented with electric motor and speed reducer which can provide peak torque of 40 N·m. This power combination is also back-drivable with extremely low friction. For rigid exoskeleton, multi-DOF mechanism helps to ensure the comfort of wearing [33]. Three connecting mechanisms, including waist part, thigh part, and crus part, are specially designed to ensure comfortable wearing. The waist support functions to transfer the weight of powered joint to the waist and to restrict the powered joint from sliding down which would give rise to its misalignment with knee joint. The battery and the control pack are also fixed to waist support through quick-release mechanism. In addition, a rotary adjustable mechanism of waist part is designed to enable quick adjustment to the individual's waist size, which is shown in Figure 1(c). A 3-DOF adjusting mechanism is specially designed for the crus part to allow adjustments according to the leg characteristics of different individuals, as is illustrated in Figure 1(d). Moreover, an IMU is attached to the waist part through a soft brace on the healthy side to collect the gait data of that.

The electrical frame of GRTR is illustrated in Figure 2. The whole electrical system is comprised of core controllers, drive unit, sensors, and power units. Two STM32F7-series microcontroller units (MCU) are utilized as the controller, one in charge of collecting the sensor data, controlling the motor, and the other one is a coprocessor for recognizing intention of the wearer with BPNN. The drive unit for knee joint is composed of brushless direct current motor and harmonic reducer integrated with encoder and torque sensor. To capture the joint information, three IMUs are integrated: one for the hip joint of the healthy side (integrated with soft brace), one for the hip joint of the hemiplegia side (embedded in powered joint shaft), and the last one for waist posture (integrated in the waist support). All the electric components communicate with MCU through the Controller Area Network.

### 2.2. Active Control Architecture

A complete gait cycle for knee joint consists of support phase and swing phase [34], as is shown in Figure 3. It usually begins with the heel striking the ground and ends with the heel striking the ground again. The joint angle varies with the process of gait phase. The objective is to recognize current walking pattern and provide corresponding joint assistance.

Based on the objective, the control architecture mainly consists of intent recognition module and flexible interaction module, as shown in Figure 4. An improved gait synchronizer driven by AFO and BP neural networks is designed for gait features detection. Two AFOs are utilized to learn gait features from hip joint of healthy side and hemiplegia side, respectively. The BPNN is cascaded with the AFOs to improve generalization of gait detection. Trained with gait data of healthy people and hemiplegia patients, the BPNN improves the gait pattern recognition performance. Then, walking states recognized by the gait detection algorithm are transmitted to the flexible interaction module. The reference assistive torque is generated according to torque database with the estimated gait phase and walking states. Finally, through the low-level direct force controller, the ideal force tracking performance is achieved to ensure the flexibility and walking assistance.

### 2.3. Intention Recognition

#### 2.3.1. AFO

Gait is a periodic motion and therefore can be learned through AFO. Based on the Hopf oscillator in [35], the differential equation of the adaptive model is described as follows:

(1) $$\begin{array}{c} \left\{\begin{array}{c} {\dot{x}}_{h}=\alpha \left(\mu^{2}-r_{h}^{2}\right)x_{h}-\omega_{h}y_{h}+\varepsilon F_{h}\\ {\dot{y}}_{h}=\alpha \left(\mu^{2}-r_{h}^{2}\right)y_{h}+\omega_{h}x_{h}\\ {\dot{x}}_{p}=\alpha \left(\mu^{2}-r_{p}^{2}\right)x_{p}-\omega_{p}y_{p}+\varepsilon F_{p}\\ {\dot{y}}_{p}=\alpha \left(\mu^{2}-r_{p}^{2}\right)y_{p}+\omega_{p}x_{p}\\ \varphi =\tan^{-1}\left(y/x\right) \end{array}\right., \end{array}$$

where *x* and *y* are the state variables in phase space and $r=\sqrt{x^{2}+y^{2}}$. The subscripts *h* and *p* stand for healthy and hemiplegia side. *μ* with *μ* > 0 represents the radius of limit cycle and controls oscillator amplitude. *ω* stands for the oscillator intrinsic frequency, and *φ* is the phase angle. The oscillator frequency *ω* will converge to the gait frequency, and phase *φ* corresponds to the gait phase. *α* represents the attraction coefficient of the limit cycle and is set as *α* = 0.5. The coupled periodic force *F* acts as the teaching signal, and *ε* is the coupling constant with value 8. The input periodic force *F* is the captured hip joint data. The oscillator has a stable harmonic limit cycle when *F* = 0. Small perturbations (*ε* > 0) only change the form and time scale of the system without the general behavior. For the adaption to the gait pattern, the system is further transformed into the following:

(2) $$\begin{array}{c} \left\{\begin{array}{c} \Delta \mu =\sigma F\;\cos\varphi =\sigma F\frac{x}{x^{2}+y^{2}}\\ \Delta \varphi =-\sigma \frac{F}{r}\sin\varphi =-\sigma F\frac{y}{x^{2}+y^{2}}\\ \Delta \omega =-\frac{\sigma }{\Delta T}F\frac{y}{x^{2}+y^{2}} \end{array}\right., \end{array}$$

where *σ* is the coefficient determining the convergence rate. Δ*T* represents system sampling time. The estimated gait phase angle is continuous and periodic, which indicates that the adaptive law is effective on frequency and phase learning.

The hip joint is the basic part of lower limb to generate gait motion. Therefore, the gait information of hip joints is utilized as the reference to predict hemiplegia side's gait intention. The kinematic data are captured from the aforementioned IMUs on the two sides. The angle information in the sagittal plane is then extracted as the inputs of two AFOs. The learned gait frequency and phase from hip joints are then imported into BPNN to recognize the knee motion.

#### 2.3.2. BPNN

The BPNN is a supervised learning method of which the output is forward-propagated and the errors is transmitted by back propagation. It has the advantages of flexible nonlinear modeling capability and strong adaptability. In addition, there is no need of huge computing resources for the trained BPNN to run in real-time, which is beneficial for the miniaturization of the system. Therefore, BPNN can be applied to establish the model between the kinematic data and gait information. Cascaded with the established AFOs, the BPNN here is to improve the gait intention recognition performance from the point of amplitude and circumstances of stroke patients.

Based on the integrated sensors in GRTR, a host of data can be collected and processed in real-time. After plenty of data analysis, those signals which have significant changes or distinctive characteristics are selected as the input of BPNN. A total of 19 signals from six parts are finally included: (1) thigh of hemiplegia side, pitch and roll angle and angular velocity in the sagittal and coronal planes; (2) waist, roll angle; (3) thigh of healthy side, same with hemiplegia side; (4) target knee, angle, angular velocity, and torque; (5) AFO output, gait frequency and phase for healthy and hemiplegia sides; and (6) last result from BPNN, current gait and next possible gaits 1 and 2. In addition, a low-pass filter with 20 Hz cutoff frequency is utilized to reject noise.

The modified BPNN is illustrated in Figure 5. There are two hidden layers in this BPNN, the first hidden layer has 30 nodes with sigmoid functions, and the second layer has 15 nodes with linear functions. And the output nodes are also with linear functions.

Apart from the the current gait, two extra possible gaits are also constructed as the outputs of BPNN, which are the next gait 1 (the gait with higher probability) and the next gait 2 (the gait with lower probability). The output next gait 1 and gait 2 focuses on possible changes of current gait according to the input data. Recognition in advance could improve the accuracy of current gait and reduce the possibility of wrong assistance.

In order to improve the recognition performance of BPNN, extensive data collection on healthy people and stroke patients has been conducted. About 1,000 data sets have been collected, each lasting at least for 5 min. Ninety percent of the data was chosen randomly as the training samples and 10% as the verification samples. In the training process, an Adam optimizer was used, and the learning rate was 0.004. After training, the determined parameters have been translated into the real-time system in Figure 2.

## 3. Experiments

### 3.1. Experimental Protocols

Preliminary validation tests on three stroke patients were conducted, and all three participants were at Stage VI of Brunnstrom recovery stage (BRS). Patients with improved motor function were recruited in consideration of safety and progressive research. Written consent was obtained from all participants. This study was carried out in accordance with the recommendations of guidelines from the Institutional Review Board approval of the Seven Affiliated Hospital of Sun Yat-Sen University (JS-2021-005-01). Detailed information of the participants can be found in Table 1.

Two series of ground-walking tests were conducted for each participant in consideration of comparison, as is shown in Figure 6. The kinematic and biomechanical data were collected using IMUs (Xsens dots) and EMG sensors (Pico EMG, Cometa) to evaluate the effectiveness of recognition and assistance. The test without wearing the knee exoskeleton came first before the test with assistance. Two exoskeletons, aiming at right and left sides, respectively, were utilized for specific participant. Participants were asked to complete six round trips within experimental site constraints. It should be noted that every participant was given several minutes to adapt to GRTR before tests with assistance. A 5-min break was taken between tests to avoid muscle fatigue. All the participants were accompanied with operator and therapist to guarantee safety. The collected data were processed after all the tests were completed.

### 3.2. Result Analysis

#### 3.2.1. Kinematic Data

To evaluate the performance of the proposed intent recognition algorithm, indexes regarding recognition accuracy and detection delay were used to assess the differences between desired knee trajectories and real-time trajectories generated by recognition [31]. To make reasonable and reliable evaluations of recognition performance, the root-mean-square error *δ*_*r*_ and peak error *δ*_*m*_ between desired gait pattern and recognized gait pattern, calculated in Equations (3) and (4) respectively, were selected:

(3) $$\begin{array}{c} \delta_{r}=\sqrt{\frac{1}{N}\sum_{i=1}^{N}{\left(u-\overset{―}{u}\right)}^{2}}, \end{array}$$

(4) $$\begin{array}{c} \delta_{m}=\max\left(u-\overset{―}{u}\right), \end{array}$$

where *u* is the recognized knee trajectory and $\overset{―}{u}$ is the desired knee trajectory. To evaluate whether the knee pattern is detected in time, the prediction time for knee trajectory of each phase of gait was calculated by *T*_*d*_ = *t*_*r*_ − *t*_*p*_. *t*_*r*_ is the moment when a gait cycle actually starts, and *t*_*p*_ is the moment when the detection occurs. Similarly, the average time delay *T*_*a*_ and peak time delay *T*_*m*_ were calculated.

One round-trip test data of participant P1 are illustrated in Figure 7(a). This test includes two sequences of flat walking, and the gap between sequences represents the interval of turning around. The interruption of walking gait was accurately recognized without inappropriate assistance. After about two steps at the beginning of each sequence, i.e., continuous walking task, the gait and algorithm turned into a stable state. The consistency of recognition and gait rhythm, as well as rapid convergence, affirmed the performance of gait recognition algorithm.

The gait data under stable walking state of participants were selected partially for further analysis. The data over about 8 s and data of one gait cycle are shown in Figure 7(b). The swing phase and support phase of each gait cycle were recognized and depicted with black line. The predicted knee motion by AFO-BPNN (red line) had good consistency with the measured real-time knee angle (blue line). The measured knee angle at the support phase was almost constant for the reason of essential little variations from gait features and uncertainty of measurement from misalignment. But the system still generated knee angle prediction at support phase based on the trained BPNN and real-time angle at swing phase. As a consequence of this character, the predicted knee angle was larger than the measured angle at the beginning of swing phase. The gait information at swing phase was then extracted and further analyzed for verification, as is shown in Figure 7(c).

The measured angle curve occurred ahead of the predicted knee angle curve. This is because that the intent recognition of knee motion is based on the occurrence of real-time knee angle. The difference was relatively obvious at the initial swing phase. The maximal and average time delay between measured and predicted knee angle was calculated for verification, as is shown in Figure 7(d).

It should be noted that the computation intervals were selected at stable gait. The maximal time delay *T*_*m*_ = 162 ms happened for P3. This is possibly because that P3 had shorter support phase and larger flexion angular acceleration at initial swing phase. The maximal time delay for P1 and P2 is 93 and 135 ms, respectively. The average time delay for participants is below 100 ms overall.

As for the recognition accuracy, the RMSE and peak error between desired flexion pattern and predicted flexion pattern for participants are shown in Figure 7(d). The RMSE for all three participants were small. But the peak error for P3 was comparatively large, *δ*_*m*_ = 19.3°, the main causes of which could be the larger flexion angle as well as larger angular velocity. The misalignment between GRTR and lower limb at higher flexion speed or acceleration could also be the influence factor. However, the recognition accuracy was generally within a specific range.

The maximum indexes should be payed attention for more comprehensive understanding of the control strategy. However, the average time delay and angle error could reflect the global features. These average indexes of the tests were at a relatively low level, and the recognition was at an effective state.

#### 3.2.2. Biomechanics

The performance of the entire control system can be reflected by the assisting effect provided by GRTR exoskeleton, which is quantified by EMG activities [36]. Two groups of muscle activities were collected for biomechanical analysis, with and without assistance, respectively [37]. The activities of quadriceps of rectus femoris (RF), vastus medialis (VM), and vastus lateralis (VL) were investigated for the influence in respect of knee extension. The biceps femoris (BF) and semitendinosus (ST) were investigated for assistance influence in respect of knee flexion. The EMG signals were captured at a sample rate of 1,000 Hz. The EMG data were band-pass filtered between 20 and 450 Hz, rectified and low-pass filtered with 6 Hz to obtain a smooth envelop [38, 39].

The sequences of several gait cycles at stable walking state were targeted. Muscle activities of RF, VL, VM, ST, and BF were captured and processed for analyzing assistance performance. The processed envelopes of EMG were segmented by each gait cycle. Further data processing including mean value and root mean square average was conducted for relevant segmented EMG envelopes [40, 41]. Figures 8(a), 8(b), 8(c), 8(d), and 8(e) illustrated the muscle activities without and with assistance for participant P1.

The muscles regarding RF (Figure 8(a)), VL (Figure 8(b)), and VM (Figure 8(c)) were targeted for extension assistance performance. According to Figure 8(f), the changes of RMSA for these three muscles are −20.4%, 13.3%, and −30.6%, respectively. The average activation for RF, VL, and VM per gait cycle shows that the extensor without assistance mainly activated at support phase and terminal swing phase. This phenomenon corresponds with the description in reference [42]. The extensor at support phase activates to prevent knee flexion and provides support stability. As for the situation with assistance, the activation of RF and VM reduced at support phase. The increase of joint stiffness with assistance from GRTR could give rise to the activation reduction. In addition, the reduction of muscle activation around terminal swing is a result of the assistance from GRTR. It should be noted that the terminal swing phase is another activation period [42]. The activation reduction at support phase and terminal phase is also valid for VL. However, the activation for VL increased around initial swing compared the situation without assistance. It could be a result of influence on muscle activation pattern from wearing the exoskeleton. Similar results also happened for participant P2 regarding extensor. But the magnitude was lower than participant P1. As for participant P3, all the muscle activation for extensor showed synchronous reduction after wearing GRTR.

Two main flexors were selected for analysis of flexion assistance performance, i.e., the BF and ST. The flexor mainly activates around terminal stance and initial swing. The activation pattern of BF (Figure 8(d)) and ST (Figure 8(e)) for P1 conformed to this theory. The flexion assistance from exoskeleton delayed the peak of activation for P1's flexor. This is because that assistance contributed to the knee flexion and reduced requirement for voluntary activation. The magnitudes of changes for ST were not solid across participants after wearing exoskeleton. However, as is shown in Figure 8(f), the activation of BF for participants with assistance showed major reductions.

From the point of majority, the GRTR provided appropriate assistance for knee flexion and extension. The reductions of activation for main extensor and flexor proved the assistance effectiveness.

## 4. Discussions

The gait intention recognition is implemented in the unilateral exoskeleton GRTR for active control. The evaluations were conducted with three stroke patients. From the perspective of kinematic data, the algorithm could recognize patient gait with small time delay and high trajectory accuracy. Accurate gait phase recognition is critical for predicting continuous trajectory and providing appropriate assistance. For stroke patients, the gait pattern is more complex regarding to changed motion sequence. Therefore, the BPNN trained with patient data enables accurate phase recognition, which is the most important contribution of this paper. As for trajectory prediction, the average indexes with small value show the stable performance of recognition. From Figures 7(b) and 7(c), the trajectory error mainly happened at preswing and initial swing phases, especially the peak error. Larger knee angle to provide foot clearance could be the reason for peak errors happening at these phases. While at midswing and terminal swing phase, high consistence could be obtained between predicted and measured trajectory. The time delay mainly happened when gait adjustments, such as the moment of turning around. As for the biomechanics, the effectiveness is reflected in reductions of EMG activation. The extensor and flexor were investigated, respectively. The reductions not only happened at swing phase, which contributed the main knee motion, but also found at support phase. The assistive torque at support phase provides the necessary knee stiffness and thus reduced the muscle activation. Apart from reduction of activation, the assistance from GRTR also regulated the muscle activation. The activation pattern of muscles was guided to more normal gait cycles, i.e., correcting the gait of hemiplegic patients.

Although relatively fine results were obtained for the tests on three stroke patients, there are still some deficiencies for the research. The patients with lower recovery stages were not recruited. These patients could show much more complex gait patterns, such as more severe compensatory movement. The data of patients with BRS Stage V have been captured and utilized for training the BPNN. But at our preliminary tests with one patient with Stage V, the assistance for correcting the gait had influences on the original compensatory movement. Although the gait with compensatory movement is not adequate, the patients could maintain relatively stable movement. With the assistance from exoskeleton, the original compensatory movement is interrupted. The patient at the preliminary test showed instantaneously reduced capacity of movement. Therefore, the proposed algorithm would focus on the patient with lower motor functions. In addition, the number of participants is another deficiency of this paper. But the objective of this paper is to propose the recognition method and conduct preliminary verification. The standard clinical verification for long-term rehabilitation effectiveness and large groups of patients will be conducted in the future. The effectiveness evaluation will be conducted through standard assessment scales and kinematic data of gait correction.

## 5. Conclusions

This paper proposed a novel intention recognition-based assistive strategy for a unilateral knee exoskeleton. This design does not rely on an accurate human exoskeleton dynamical model or complicated EMG, EEG signals to evaluate motion; instead, the adaptive oscillators coupled with a BP neural network driven by joint angular information are presented to estimate gait frequency, phase, and amplitude. Moreover, the detected gait intention is imported as reference signals to flexion interaction module for providing appropriate assistance. Practical experiments have been carried out to verify the good performance of gait motion recognition and rehabilitation assistance. The comparative analysis of kinematics and biomechanics between walking tasks with assistance and without assistance proved the assistive effectiveness.

## Figures and Tables

**Figure 1:** Mechanical design of GRTR: (a) convenient wearing of GRTR for the user; (b) the overall structure of GRTR; (c) the waist part with adjustment mechanism; and (d) the connection part with 3-DOF adjustment mechanism for shank.

**Figure 2:** Electronic design of GRTR.

**Figure 3:** A gait cycle for knee joint.

**Figure 4:** Control architecture of GRTR. The intent recognition module consists of the adaptive oscillator and BP neural network. Recognized gait intention is imported into the following flexible interaction module to provide appropriate assistance.

**Figure 5:** The modified BPNN for gait pattern detection.

**Figure 6:** Experimental settings: (a) the test without exoskeleton and (b) the test with assistance from exoskeleton.

**Figure 7:** Gait information from tests: (a) the data of one test for participant P1; (b) the data over 8 s for P1; (c) the data over one gait cycle; and (d) the evaluation performance for all participants.

**Figure 8:** EMG activities for participants: (a–e) describe the average activities of RF, VL, VM, BF, and ST for participant P1 without assistance (red line) and with assistance (blue line). The shaded areas represent the standard error deviations, and (f) illustrates the change of RMSA for EMG activities in percentage for participants P1–P3.

**Table 1:** Participants' information.

Subject	Gender	Age	Height (cm)	Weight (kg)	Hemiplegia side
P1	Male	65	170	60.0	Right
P2	Female	34	160	55.0	Right
P3	Male	41	176	70.5	Left

## Data Availability

The raw data required to reproduce these findings cannot be shared at this time as the data also form a part of an ongoing study. The processed data are available upon request by contact with the corresponding author.
